The article "Research on Agricultural Product Traceability Technology (Economic Value) Based on Information Supervision and Cloud Computing" was published in 2022. Journal: Comput Intell Neurosci.

# Research on Agricultural Product Traceability Technology (Economic Value) Based on Information Supervision and Cloud Computing

**DOI:** 10.1155/2022/4687639

**Published:** 2022-01-30

**Authors:** Rongkuan Wang, Xi Chen

**Affiliations:** ^1^School of Business Administration, Zhongnan University of Economics and Law, Wuhan, Hubei 430073, China; ^2^Nanchang Business College of Jiangxi Agricultural University, Jiujiang, Jiangxi 332020, China

## Abstract

Traditional agricultural product traceability system adopts centralized storage, and the traceability process is solidified, which results in the low reliability of traceability results and the poor flexibility of the system. Aiming to solve this problem, blockchain technology is applied to supply chain traceability, and a supply chain traceability system based on sidechain technology is proposed. Goods management, information sharing, and product traceability in supply chain are realized through Ethereum smart contract. The sidechain technology is adopted to expand Ethereum so that it can meet the needs of practical applications. The experiment results show that the proposed system has a transaction function and information sharing function. Compared with similar trading systems, the proposed system has more advantages in throughput and security.

## 1. Introduction

ptTraceability of agricultural products refers to the forward tracing and reverse tracing of all links of the industrial chain from production to circulation of agricultural products [1]. After years of development, the traceability system of agricultural products in China is becoming perfect. However, it still has some problems, such as low reliability of traceability results and poor system flexibility. From the very beginning, the agricultural product traceability system has attracted the attention of experts at home and abroad. As early as 2002, the US Congress passed the “Bioterrorism Act” to establish the traceability system of agricultural product quality and safety [2]. So far, the community has reached a consensus on the importance of traceability of agricultural product quality and safety. The construction of relevant systems and systems has also achieved initial results, but there are still many problems in practical work.

In the context of the rapid development of industry 4.0, many new technologies have been applied in the production, management, and harvesting of agricultural products. The application of these technologies makes the production management of agricultural products more intelligent, efficient, and transparent. Among them, agricultural product traces technology also to ascend a new step. Literature [3] describes the possibility of realizing food quality testing during transportation from manufacturer to consumer. It uses a sensor remote monitoring system combined with the Internet of Things technology to propose a low-cost solution based on Internet of Things real-time food tracking and food transportation process monitoring. Although the Internet of Things technology is mature enough, the production and sales system of agricultural products involves many subjects, complicated uncertainties affecting the system, and large resource consumption for real-time monitoring with the help of sensors [4]. These will lead to difficult and inefficient management of quality and safety traceability system; especially, data storage security is still facing many challenges and problems.

In order to improve the reliability and flexibility of agricultural product traceability system, blockchain can be used to replace the traditional centralized database. It ensures the safe storage of traceability data and nonrepudiation of information source to achieve reliable traceability of agricultural products [5]. In addition, it can decouple the whole industrial chain into multiple independent links and combine them with independent channels in the super ledger into link modules. It can coordinate with the module allocation mechanism, dynamically adjust the traceability process according to the actual production, and finally realize the dynamic traceability of agricultural products. In literature [6], it is proposed to use blockchain distributed storage technology to solve the possibility of tampering or destroying data in the data storage stage by virtue of the irreversibility of blockchain.

Developed from the underlying technology of Bitcoin, blockchain is a distributed storage technology featuring decentralization, traceability, nontampering, openness and transparency, consensus mechanism, and transaction anonymity. However, compared with other industries, blockchain technology for agricultural product quality and safety traceability puts more pressure on the storage of IoT data. In order to achieve the consistency of distributed nodes, the block generation speed and transaction processing capability of blockchain are limited. Therefore, it is not possible to directly apply blockchain technology to process and store large amounts of sensor data. In order to solve the storage problem, cloud computing and cloud storage technologies are used in literature [7] to provide applications. As mentioned in literature [8], the traditional security problems still exist in cloud computing environment, and even traditional security mechanisms are no longer applicable to applications and data in cloud. In literature [9], the dual-chain structure of blockchain is proposed, which uses a chained data structure to store blockchain transaction hashes. It works with the blockchain to form double-chain storage that ensures that agricultural data cannot be tampered with or destroyed. As there are many standards involved in agricultural product traceability, effective policy control is needed for participating nodes. As the amount of data increases, the efficiency of blockchain transactions also increases. A complete public chain can no longer meet these variable needs. Compared with public chain, alliance chain has more advantages in high availability, high performance, programmability, and privacy protection. It is considered as the “partially decentralized” or “polycentric” blockchain. Alliance chain simplifies the number of nodes, which can make the system run more efficiently and cost less. It can confirm that the number of transactions per unit of time is much larger than the public chain, and it is easier to land in the agricultural product quality and safety traceability system.

There are two main problems in big data recording. The first is the issue of record speed caused by the blockchain consensus algorithm. While anyone is free to use Bitcoin's blockchain, only seven writes per second are the limit of its performance. The second is the boundary of the number of participating nodes. Even in participant-limited blockchains targeted at commercial use, the performance deteriorates dramatically when the number of participating nodes exceeds a few dozen.

In view of the problems existing in the traditional agricultural supply chain system, such as difficulties in trust transmission, opaque transaction information, and difficult information sharing, this paper proposes an agricultural products traceability system of blockchain. In the agricultural product traceability system, the performance of the blockchain is affected as the agricultural product data increases. Sidechain technology can provide some functions such as smart contracts and privacy protection on top of the main chain. These features ensure that users can use them without affecting the performance of the main chain. Therefore, in order to improve the performance of the main chain, this paper uses sidechain technology to expand the capacity of Ethereum to meet the demand of supply chain traceability information on the chain. The innovations and contributions of this paper are listed as follows:

1. Aiming to solve the problem that the traditional agricultural product traceability system has the low reliability of traceability results and poor flexibility, this paper proposes a supply chain traceability system based on sidechain technology.
2. Goods management, information sharing, and product traceability in supply chain are realized through Ethereum smart contract. The sidechain technology is adopted to expand Ethereum so that it can meet the needs of practical applications.

The structure of this paper is as follows. The traditional agricultural products traceability system is described in the next section. The current state of blockchain traceability systems is described in Section 2. Section 4 focuses on the design of an agricultural product traceability system. Section 5 presents the experiment and analysis. Section 6 is the conclusion.

## 2. Traditional Agricultural Products Traceability System

### 2.1. Traditional Traceability Mode

In 2006, China proposed the establishment of agricultural product quality and safety traceability system [10], which has achieved fruitful results after years of development. Literature [11] proposed a technical system of agricultural product quality safety traceability system of “one core, two axes, and three chains” based on the characteristics of Internet of Things technology. Literature [12] proposed the traceability chain hierarchical model of the traceability system based on the food chain. Literature [13] designed a multilateral traceability system for agricultural product quality safety in view of the decentralized and noncentralized characteristics. Literature [14] constructed a design scheme of agricultural product quality traceability system based on Fabric blockchain implementation strategy. By analyzing the typical traceability system, the traceability model of traditional agricultural products is obtained, and its structure is shown in Figure 1.

Traditional agricultural product traceability system generally centers on a centralized database. In the actual production process, the supply, planting, storage, logistics, and sales of production materials in the industrial chain are arranged in sequence. Then, the traceability data is uploaded to the centralized database. The quality supervision department supervises the quality of agricultural products by collecting information from centralized databases. Consumers send a query request to the centralized database to obtain the traceability information of purchased agricultural products.

### 2.2. Existing Problems

In the early stage of agricultural product traceability research, researchers usually focus on the full collection of traceability data and complete coverage of the industrial chain. The research on data security storage and system dynamic traceability is relatively few, which leads to the lack of reliability and flexibility of traditional agricultural product traceability system. Some researchers apply blockchain technology to the traceability of agricultural products but seldom optimize the traceability process and system structure by combining the characteristics of both. While the traceability results obtained are reliable, there is still a lot of room for improvement in the flexibility of the system.

Traditional agricultural product traceability system stores data in a centralized database, which brings a series of data security problems. This reduces the credibility of the traceability system for agricultural products. Traditional traceability systems usually trace specific agricultural products in a narrow range. The limitation of traceability objects and production process leads to the solidified transaction processing process of the traceability system. It cannot dynamically adjust the sequence of production link combination according to the actual production scene, which is not conducive to system function expansion and upgrade. These factors lead to poor flexibility of the traceability system.

## 3. The Current State of Blockchain Traceability Systems

### 3.1. Supply Chain Traceability System Based on Blockchain

At present, there are many researches and applications in academia and industry to realize supply chain traceability by using blockchain. Literature [15] applied blockchain to drug supply chain traceability system. It used affiliate link technology and quick response (QR) encrypted codes to establish full-chain traceability for drugs from manufacturer to seller. Literature [16] proposed a new two-step block-out method and designed a joint distributed ledger CoC (supply chain on blockchain) based on this method for supply chain management system. The experimental results show that the two-step block extraction method has good performance, which is faster, more efficient, and safer. Literature [17] used blockchain technology to enhance the elasticity of the supply chain and studied the basic framework of blockchain and its underlying technology. It analyzed the various risks facing the current supply chain and described the specific application scenarios of blockchain technology in the supply chain.

The above literature involves the research of supply chain traceability system but generally does not involve the underlying blockchain platform. In addition, it lacks running and testing on the blockchain. In industry, food industry giants are using blockchain technology to reform the food supply chain. Walmart, IBM, https://www.JD.com, and Tsinghua University set up a safe food blockchain traceability alliance. It uses blockchain technology to track the food supply chain and build safe tables. Among them, Hyperledger developed by IBM, as a kind of underlying blockchain technology, has been widely applied in various fields of supply chain by major companies. In China, Tmall International products use ant blockchain independently developed by Alibaba for cross-border product traceability, which greatly increases the security of imported goods. The Institute of Intelligent Supply Chain Management of Tsinghua University cooperated with Yonghui Supermarket to use steel gash to trace the numbers of Xingcheng Turbot fish. It achieves one yard per fish to ensure food safety and has been promoted to more than 10 kinds of fresh products. Jingdong Y Business Department launched the Baas platform of “Zhizhen Chain” to realize the traceability of some commodities in Jingdong supermarket by using this platform.

At present, alliance chain technology is basically used in supply chain traceability projects. An affiliate chain is a blockchain network that allows only certain group members and limited third-party access. Because of the access mechanism, the small number of nodes, the use of a high-performance consensus algorithm, and other reasons, the alliance chain usually has higher transaction performance than the public chain. Moreover, the alliance chain can provide queries and other functions to the third party in the form of open API, which is more friendly to supervision. Therefore, it is called “Blockchain 3.0,” which flaunts the future development direction of blockchain. The demand and background of the supply chain are consistent with the alliance chain: the members of the supply chain are limited and fixed. The up-chain of supply chain information requires faster transaction speed and lower transaction cost. Supply chain traceability needs the supervision of relevant departments. Therefore, alliance chain technology is suitable for supply chain traceability system. Currently, one of the more active and recognized open-source consortium projects is Hyperledger Fabric developed by IBM. Most blockchain platforms are improved and encapsulated based on Hyperledger.

However, relevant researches show that there are many difficulties in the realization of the alliance chain. Its main bottleneck lies in the weak financial strength of small and micro enterprises, that is, they are unable to maintain the servers required by the alliance chain. Consensus nodes are typically deployed in large enterprises and some third-party organizations. Small and microenterprises in the supply chain generally only have terminal or Internet of Things acquisition devices and do not configure a consensus server. This leads to the imbalance of consensus rights in the alliance chain and the failure of consensus strategies due to too few consensus nodes. In actual deployment, core enterprises gradually deploy consensus nodes in the same consensus domain. Docker container technology is used to generate four nodes on the same server for consensus, and other enterprises in the supply chain use clients to access the alliance chain. This operation saves costs and facilitates small applications and early commissioning. However, it violates the original intention and principle of the alliance chain and cannot play the role of the alliance chain. This system is developed based on Ethereum smart contract to realize supply chain traceability in a decentralized way to save costs for enterprises on the chain.

### 3.2. Sidechain Technology

To implement supply chain traceability on Ethereum, transaction costs must be considered. Suppliers, processors, and distributors shall chain raw material information, product processing information, and product sales information, respectively. This data can put a lot of pressure on the Ethereum main network and lead to high transaction fees, as well as high confirmation delays. In this paper, sidechain technology is used to expand Ethereum to meet the demand of supply chain traceability information.

The sidechain technology was first used in the expansion of Bitcoin. It is a protocol that allows Bitcoin to be safely transferred to other blockchains and safely returned to the main Bitcoin chain from other blockchains. The protocol moves some frequent, small transactions onto the sidechain. This not only improves the efficiency of Bitcoin's main network but also significantly reduces transaction fees. Therefore, the deployment of the corresponding sidechain technology on Ethereum can reduce the pressure on the main network of Ethereum and improve transaction efficiency. At present, common Ethereum sidechain protocols include Loom Plasma Chain and Snarky. The Loom PlasmaChain is a high-performance DPoS (delegated proof of stake) sidechain that implements the Plasma Cash framework model. It can gain security endorsement from Ethereum's underlying network, allowing users to enjoy the high-performance consensus of DPoS algorithms when using tokens supported by ERC 20 and ERC 721. Snark sidechain solution can expand Ethereum network transaction capacity up to 17000 TPS as a kind of down chain expansion. Snark allows users to transfer tokens and ETH outside Ethereum.

In the existing studies, the sidechain expansion schemes of Bitcoin and Ethereum only include token transfer. Token transactions are transferred to the sidechain for higher throughput and lower handling fees. This paper constructs a sidechain model of user data transfer to provide an expansion scheme for supply chain traceability information so that the supply chain traceability system based on Ethereum can be applied to the actual production.

## 4. The Design of Agricultural Product Traceability System

### 4.1. System Architecture

In this paper, aiming at the shortcomings of the existing agricultural supply chain traceability scheme, Ethereum and smart contract are used to design and implement a supply chain traceability system based on sidechain technology. Its architecture is shown in Figure 2. The smart contract module contains the business logic of the system. It deploys this module on the sidechain, which can greatly increase the efficiency of Ethereum usage, reduce transaction confirmation time, and reduce transaction costs. The data synchronization module is responsible for processing each batch of transaction data and using the Merkle tree algorithm to obtain the transaction hash value. It synchronizes the hash value to Ethereum for locking. When consumers and regulators query, the data synchronization module can be used for calculation and verification to prevent data tampering.

In the blockchain supply chain traceability system network, enterprises such as suppliers, manufacturers, and distributors use the Internet of Things collection equipment to collect product information. It generates raw data, uses a terminal for data processing, and sends it to a sidechain server. The sidechain server is maintained by the core enterprise and runs the Ethereum sidechain process. It connects to the Ethereum public chain for data storage. The supervisor and the user use PC and mobile device, respectively, to access the sidechain server and verify the authenticity of the data on the Ethereum public chain.

### 4.2. Contract Design

There are five types of participants in the supply chain traceability system based on blockchain. As a raw material supplier, the supplier is the source of a batch of product information traceability. It requires the creation of an initial file and traceability number for the raw material. The manufacturer processes and distributes the raw materials and is the source of information for the smallest selling unit of the product. It needs to assign batch numbers and QR codes to traceability products, to achieve one code for one thing. Dealers buy from manufacturers and sell through different channels. It needs to provide information on warehousing, logistics, and so on. The supervisor supervises the production, circulation, and operation of commodities. Consumers can scan the QR code to view the traceability information of the whole life cycle of the product. The relevant operations and processes of participants on smart contracts are shown in Figure 3.

Smart contract includes the following five functions:

1. User registration. Since the public chain itself has no identity authentication mechanism, it needs to realize user access through smart contract. Companies in the same supply chain need to agree on a number before entering information. The user is registered by executing the userRegister() function. This number groups these companies into a user group, and only the users in the group can add traceability information to the products on the chain. The pseudocode of the userRegister() function algorithm is shown in Algorithm 1.
2. Input raw materials. As the information source of the supply chain, suppliers need to use the Internet of Things equipment to collect the data of the production environment, production cycle, and the person in charge of operation of raw materials. The rawRegister() function is then used to chain up the data, create an initial file for the raw material, and assign the raw material lot number. For example, a batch of raw material traceability file is modeled as <rawID, rawName, rawFac, produceTime, rawInfo>. The rawRegister() algorithm pseudocode is shown in Algorithm 2.
3. Product production. The manufacturer processes the raw materials provided by the supplier to produce the minimum selling unit of the commodity. In this link, product files based on traceability source code are formally established and provided to consumers in the form of two-dimensional code for inquiry. The manufacturer needs to call the newProduct() function to integrate the raw material information. It can also write URLs to production environment, production video, and other large files in the product_info field.
4. Product distribution. This feature records the circulation of products, helps consumers to check the source of goods, and helps manufacturers to prevent the diversion of goods. After handling the goods, the distributor or logistics enterprise uses the product_deal() function to add the distribution information to the goods. Because one or more handling enterprises exist, product information is stored in the structure using the dynamic array Bytes32 retailerNames. Since the code logic is like raw material entry, the pseudocode of the production and distribution functions will not be described here.
5. Supervision and inquiry. Consumers can query the traceability information of the batches to which the goods belong, and supervisors have higher authority when querying the goods. In the query function, the identity of the inquirer is first authenticated, and the batch file of the product is returned to the inquirer after passing.

### 4.3. Data Synchronization and Verification

After the product traceability information is stored on the sidechain, the Merkle tree algorithm is used for hash locking, and the resulting Merkle Root is synchronized to the Ethereum main chain. Merkle Root changes when traceability information is tampered with.

After a round of trading, the information uploaded by suppliers, manufacturers, distributors, and other nodes in the sidechain is taken as the leaf nodes of the Merkle tree to calculate its hash value. If there are multiple suppliers or resellers, the information from the different nodes is processed as leaf nodes. After obtaining several hashes (H1, H2,…), perform pairwise hash operation on (H1, H2,…) to obtain the hash value. The pseudocode of the Merkle tree algorithm is shown in Algorithm 3.

Bind Merkle Root to the product batch number and synchronize it to the Ethereum main chain, which can be used as the traceability verification code of this batch of products. After the user queries the product traceability information, the same method is used to obtain Merkle Root. This can be compared to a reliable value on Ethereum to determine whether the traceability information for the product has been tampered with. Once the data is incorrect, regulators can use the Merkle tree algorithm to locate more quickly which branch the tampered data came from. Then, the accountability can be investigated in the corresponding supply chain links.

### 4.4. System Business Process

The business process of supply chain traceability system designed in this paper is shown in Figure 4. Goods are traced back to their original raw materials. The process from rough machining by the supplier to finish machining by the manufacturer can be traced. The process from sales channels to consumers can also be traced back. All information can be tracked in an all-round, multiangle, and wide field. In this way, the origin and destination of products can be traced.

## 5. Experiment and Analysis

### 5.1. Fault Tolerance Test of Trading System

The ability to operate stably when a system is attacked by a malicious node is called system fault tolerance. Therefore, the probability of a certain number of malicious nodes successfully destroying the normal operation of the system is taken as an index to evaluate the fault tolerance performance of the system. Considering the experimental effect and equipment performance, the number of nodes in the supply chain system was set to 50, and the number of malicious nodes gradually increased from 0 to 30. The successful rate of attack of malicious nodes in different states is obtained through several experiments under different number of malicious nodes.

In the supply chain system, the core enterprise will check the qualification of the enterprise applying to join the supply chain. Therefore, the probability that the number of malicious nodes exceeds 1/3 of the total number of nodes is low. At this time, according to Figure 5, the attack success rate is very low. The system has a high fault tolerance performance under the current conditions, but considering malicious attacks outside the system, the system fault tolerance performance needs to be further improved.

### 5.2. Throughput Analysis of Trading System

Transaction Per Second (TPS) is used to evaluate system throughput. The transaction system undertakes the transaction function of the supply chain and has certain requirements on the real-time performance of the system. This paper analyzes the throughput of the supply chain transaction system through experiments, which provides a good foundation for system upgrade and deployment. The number of nodes of the trading system was taken as a variable in the experiment, and the number of nodes increased from 0 to 70. The experiment was repeated under different number of nodes. Finally, the TPS value of various nodes is used as the indicator of system throughput in various states.

It can be seen from Figure 6 that when the number of nodes is 5–45, the throughput of the transaction system rises with the increase of the number of nodes, and the upward trend remains basically unchanged. The throughput of the system in this paper is still small, even in the experimental environment where the operating environment is stable, and the interaction content is simple. There is still a gap between this and the huge data transaction demand of the supply chain. Therefore, according to the actual demand of the supply chain, multichain and layered technologies will be combined to optimize the system architecture in the subsequent research. At the same time, the consensus algorithm is improved by using the advantages of the alliance chain and supply chain system to improve the consensus efficiency and increase the system throughput.

### 5.3. Comparison of Transaction Throughput

The throughput is an important indicator to evaluate the transaction system and blockchain system. Therefore, the throughput of the transaction system in this paper is compared with that of the transaction system in literature [18–20]. In the experiment, the number of nodes of the trading system was taken as a variable, and the number of nodes increased from 0 to 60. The experiment was repeated under different number of nodes, and the average value of TPS under different states was obtained as shown in Figure 7.

According to the experimental results, when the number of nodes is less than 40, the transaction system in this paper has certain advantages in throughput performance. However, the throughput of the transaction system in literature [18, 19] continues to rise and does not decline when the number of nodes reaches 60. Therefore, when the number of nodes in the transaction system is small, the transaction system in this paper has certain advantages in throughput performance. However, the system throughput peak value is small, which has a certain gap with the actual application demand of the supply chain system, and the system throughput performance has a large space to improve.

## 6. Conclusion

Traditional agricultural product traceability system is generally centered on a centralized database, which leads to the difficulty of traceability and inflexibility of the system. While blockchain technology is in the development stage, how to break through the technical bottleneck of blockchain and better apply it to the production of agricultural products has become the focus of the industry. In order to promote the cooperation between enterprises in the supply chain and improve the efficiency of supply chain cooperation, this paper designs a chain traceability system of agricultural products based on sidechain technology. It provides a trusted platform for data sharing, which is independent of third parties. The experimental results show that the system combines sidechain technology with supply chain traceability, and it provides an expansion scheme for nontransfer transactions. The future work is to compare and analyze different sidechain protocols and select the high-performance sidechain technology that is more suitable for supply chain traceability system to improve the transaction performance of the system.

## Figures and Tables

**Figure 1:** Structure of traceability model for traditional agricultural products.

**Figure 2:** Supply chain traceability system architecture.

**Figure 3:** Operation flow of smart contract.

**Figure 4:** Business process of the traceability system.

**Figure 5:** Success rate of trading system attack.

**Figure 6:** The throughput of the transaction system under different number of nodes.

**Figure 7:** Throughput comparison of the trading system.

**Algorithm 1:** userRegister() function.

**Algorithm 2:** rawRegister() function.

**Algorithm 3:** Merkle tree algorithm.

## Data Availability

The labeled dataset used to support the findings of this study is available from the corresponding author upon request.
